RETRACTED

# miR-223-3p alleviates TGF-β-induced epithelial-mesenchymal transition and extracellular matrix deposition by targeting SP3 in endometrial epithelial cells

**DOI:** 10.1515/med-2022-0424

**Published:** 2022-03-11

**Authors:** Yanling Chen, Dongyan Sun, Di Shang, Zhihe Jiang, Pan Miao, Jian Gao

**Affiliations:** Department of Obstetrics and Gynecology, School of Medicine, Wuhan University of Science and Technology, Wuhan 430072, Hubei, China; Department of Gynecology, Maternity and Child Health Care Hospital of Hubei Province, 745 Wuluo Road, Wuchang District, Wuhan 430000, Hubei, China; Yangtze University Health Science Center, Jingzhou 430199, Hubei, China

**Keywords:** intrauterine adhesion, miR-223-3p, TGF-β, SP3, endometrial epithelial cells

## Abstract

Intrauterine adhesion (IUA) is the clinical manifestation of endometrial fibrosis. The dysregulation of microRNAs (miRNAs) has been confirmed to implicate in a diversity of human diseases, including IUA. Nevertheless, the specific function of miR-223-3p in IUA remains to be clarified. Reverse transcription quantitative polymerase chain reaction analysis displayed the downregulation of miR-223-3p in IUA tissues and endometrial epithelial cells (EECs). Results from wound healing assay, Transwell assay and western blotting showed that TGF-β facilitated the migration and invasion of EECs and induced epithelial-mesenchymal transition (EMT) process as well as extracellular matrix (ECM) deposition. Overexpression of miR-223-3p in EECs was shown to suppress the effects induced by TGF-β. Bioinformatics analysis and luciferase reporter assay revealed the binding relation between miR-223-3p and SP3. SP3 was highly expressed in IUA and its expression was inversely correlated with miR-223-3p expression in IUA tissue samples. Additionally, upregulation of SP3 reversed the influence of miR-223-3p on the phenotypes of EECs. In conclusion, miR-223-3p alleviates TGF-β-induced cell migration, invasion, EMT process and ECM deposition in EECs by targeting SP3.

## 1 Introduction

Intrauterine adhesion (IUA), characterized by endometrial fibrosis, is a uterine disease caused by trauma, infection, inflammation and other factors [1]. Patients with IUA may suffer from pelvic pain, abnormal menstruation, recurrent abortion, infertility and pregnancy complications [2,3]. The main approach adopted for IUA treatment is transcervical resection of adhesions via hysteroscopy followed by re-adhesion prevention [4,5]. However, the recurrence rate after treatment is still high. It was reported that the recurrence rate of mild and moderate IUA is approximately 30% and that of severe cases is as high as 62.5% [6,7]. Hence, it is of great significance to find a better method to prevent adhesion formation.

RETRACTED

Endometrial fibrosis is the primary pathological characteristic of IUA [8]. It has been indicated that epithelial-mesenchymal transition (EMT) of endometrial epithelial cells (EECs) plays an indispensable role in endometrial fibrosis [9]. In EMT process, cells lose the epithelial features and gain migratory and invasive mesenchymal properties [10]. Furthermore, extracellular matrix (ECM) deposition is another important pathological change in IUA which results in endometrial fibrosis [11]. ECM deposition is characterized by enhanced levels of protein markers, such as alpha smooth muscle actin (α-SMA) and type I collagen (collagen I) [12]. Transforming growth factor-beta (TGF-β) is a multifunctional cytokine which has significant effects on various biological processes, including cell proliferation, invasiveness and differentiation [13,14]. Importantly, TGF-β was reported to be closely associated with EMT and ECM [15,16].

MicroRNAs (miRNAs) are noncoding RNAs of 18–25 nucleotides that regulate over 60% of protein-coding genes [17,18]. Abnormal expression of miRNAs is strongly related to a variety of human diseases, including IUA [19]. For example, miR-326 suppresses endometriosis in IUA by modulating TGF-β1/Smad3 pathway [20]. miR-466 interacts with NUS1 in IUA in a rat model by regulating AKT/NF-kB signaling pathway [21]. Importantly, miR-223-3p is aberrantly expressed in many diseases. miR-223-3p acts as a regulator in the pathogenesis of multiple disorders, associated with fibrosis, inflammation and other clinical features [22] Dysregulation of miR-223-3p plays a key part in various biological processes. For example, in benign prostatic hyperplasia, miR-223-3p overexpression facilitates cell proliferation, migration and EMT by targeting MAP1B [23]. Nevertheless, the detailed function and mechanism of miR-223-3p in IUA remain obscure.

SP3 transcription factor, belonging to a family of SP1 related genes, encodes a protein that acts as a bifunctional transcription factor to either stimulate or repress the transcription of numerous genes [24]. SP3 was reported to be downregulated in stromal cells of secretory in human endometrium [25]. Moreover, overexpression of SP1 and SP3 stimulates the promoter activity of HSD17B2 in EECs [26]. Based on the above evidence, it was hypothesized that miR-223-3p might exert its effect by SP3.

This study aims to reveal the role and mechanism of miR-223-3p in the dysfunctions of EECs, which might develop a novel therapeutic target for treating IUA.

## 2 Materials and methods

### 2.1 Clinical specimens

Twenty pairs of endometrial tissues were collected from patients with IUA (4 mild cases, 10 moderate cases and 6 severe cases) or infertility who underwent hysteroscopy in Maternity and Child Health Care Hospital of Hubei Province from August 2019 to December 2020. The prognostic classification and adhesion scoring of IUA was based on the American Fertility Society Classification of 1988. The age of all participants at the time of entry ranged from 20 to 40 years. Endometrial tissues from all participants were obtained in the late proliferative phase based on 15–18 mm size of dominant follicle (transvaginal ultrasound scan) and a plasma progesterone level <5.5 nmol/L. The acquired endometrial tissues were immediately stored in liquid nitrogen at −80°C for further experiments. Written informed consent was obtained from all patients. The study was approved by the Ethics Committee of Maternity and Child Health Care Hospital of Hubei Province.

RETRACTED

### 2.2 Cell culture and transfection

EECs were obtained from Ribobio (Guangzhou, China). Cells were cultured in Dulbecco’s Modified Eagle’s Medium (DMEM, Corning, NY, USA) containing 10% fetal bovine serum (FBS, Corning), 100 U/mL penicillin (Corning) and 100 µg/mL streptomycin (Corning), and maintained in a humidified incubator at 37°C with 5% CO_2_. TGF-β (5 µg/mL) was added to the medium and cultured for 24 h to stimulate the cells [27]. For cell transfection, miR-223-3p mimics (or NC mimics) and pcDNA3.1/SP3 (or control pcDNA3.1) were transfected into EECs to overexpress miR-223-3p and SP3, respectively. All plasmids were constructed by Ribobio. Cell transfection was achieved using Lipofectamine 2000 (Invitrogen, Carlsbad, CA, USA). After 48 h, reverse transcription quantitative polymerase chain reaction (RT-qPCR) was used for the detection of transfection efficiency.

### 2.3 RT-qPCR

Total RNA was isolated from EECs using TRIzol reagent (Invitrogen). Reverse transcription of 2 µg RNA into cDNA was conducted using ReverAid First Strand cDNA Synthesis Kit (Thermo Scientific, Waltham, MA, USA). RT-qPCR was implemented with GoTaq qPCR Master Mix Kit (Applied Biosystems, Foster City, CA, USA). The relative expression of miR-223-3p was normalized to U6 and calculated by the 2^−ΔΔCt^ method. Primer sequences are provided as follows:

hsa-miR-223-3p

Forward: 5′-GCGCGTGTCAGTTTGTCAAAT-3′

Reverse: 5′-AGTGCAGGGTCCGAGGTATT-3′

U6

Forward: 5′-CTCGCTTCGGCAGCACA-3′

Reverse: 5′-AACGCTTCACGAATTTGCGT-3′.

### 2.4 Western blotting

EECs were lysed with RIPA lysis buffer (Beyotime, Shanghai, China). The protein concentration was measured by a BCA assay kit (Beyotime). Protein samples were separated on 10% SDS-PAGE gel electrophoresis and transferred to polyvinylidene fluoride membranes (Millipore, MA, USA). The membranes were blocked with 5% skimmed milk before incubation with the following primary antibodies: anti-E-cadherin (ab40772, 1:10,000), anti-N-cadherin (ab76011, 1:5,000), anti-Vimentin (ab92547, 1:1,000), anti-α-SMA (ab32575, 1:1,000), anti-collagen I (ab34710, 1:1,000), anti-β-actin (ab6276, 1:5,000), anti-FBXW7 (ab192328, 1:1,000) and anti-SP3 (ab227856, 1:3,000) (all from Abcam, Cambridge, CA, USA) overnight at 4°C. Afterwards, the membranes were further incubated with the secondary antibody (Abcam) for 2 h at room temperature. The signals were visualized with an enhanced chemiluminescence kit (FDbio science, Hangzhou, China) and quantified with ImageJ software (GE Healthcare, Beijing, China).

RETRACTED

### 2.5 Wound healing assay

To measure the migrative abilities of EECs, transfected cells were plated into 6-well plates until confluency to 70%. Afterwards, a standard 10 µL pipette tip was utilized to scratch the center of the plates. The cell movement was recorded at 0 and 24 h by ImageJ software (National Institutes of Health, Bethesda, MD, USA). Healed wound percentage was calculated as:

\text{(Original}\hspace{.25em}\text{wound}\hspace{.25em}\text{width}-\text{Current}\hspace{.25em}\text{wound}\hspace{.25em}\text{width)/(original}\hspace{.25em}\text{wound}\hspace{.25em}\text{width)}\text{.}]

### 2.6 Transwell assay

The migration of EECs was examined in 24-well plates using chambers coated with Matrigel (BD Biosciences, Bedford, MA, USA). After pre-treatment, cells were inoculated (1 × 10^5^ cells/well) into the upper chambers containing serum-free medium, and the lower chambers were added with DMEM containing 10% FBS. Cells were cultured at 37°C with 5% CO_2_ for 24 h. After that, noninvasive cells were removed with a cotton swab. The invasive cells were fixed in 4% paraformaldehyde, stained with 0.1% crystal violet and imaged using a phase-contrast microscope (Olympus, Tokyo, Japan).

### 2.7 Luciferase reporter assay

The binding site between miR-223-3p and SP3 3′UTR was predicted with TargetScan (http://www.targetscan.org/vert_71/). Phusion Site-Directed Mutagenesis Kits (Thermo Fisher Scientific, Waltham, MA, USA) were used to mutate the predicted binding site of miR-223-3p on SP3 3′UTR. Wild type or mutant SP3 3′UTR fragment was synthesized and subcloned into pGL3 vectors (Promega, Madison, WI, USA) to construct SP3-Wt or SP3-Mut vectors, respectively. EECs were transfected with above plasmids and miR-223-3p mimics (or NC mimics) using Lipofectamine 3000 (Invitrogen). A dual luciferase reporter assay kit (Invitrogen) was used for the detection of luciferase activity.

### 2.8 Statistical analysis

All data were analyzed using SPSS 20.0 software (Promega) and are presented as the mean value ± standard deviation (SD). Each experiment was implemented at least three times. Student’s *t*-test was used for difference comparisons between two groups, while analysis of variance (ANOVA) was used for comparisons among many groups followed by Tukey’s *post hoc* analysis. The expression correlation between miR-223-3p and SP3 in IUA tissues was identified using Pearson analysis. *p* < 0.05 was regarded to be significant.

RETRACTED

## 3 Results

### 3.1 TGF-β induces EMT process, ECM deposition and miR-223-3p downregulation

First, we examined the impacts of TGF-β in EECs. As displayed by wound healing assay, the percentage of healed wound was obviously raised by TGF-β (Figure 1a). Likewise, the number of migratory and invaded cells were increased by TGF-β, as revealed by Transwell assay (Figure 1b). The above results suggested that TGF-β strengthened the migratory and invasive capabilities of EECs. Moreover, western blotting was utilized for the measurement of EMT-associated protein and ECM protein levels. As expected, TGF-β reduced the level of E-cadherin, and enhanced the levels of N-cadherin, Vimentin, α-SMA and collagen I (Figure 1c), suggesting that TGF-β induced EMT process and ECM deposition in EECs. Additionally, miR-223-3p level was notably reduced in TGF-β group in comparison to the control group (Figure 1d). As shown by RT-qPCR, miR-223-3p was downregulated in the endometrial tissues of IUA patients compared to that in normal tissues (*N* = 20 pairs) (Figure 1e).

**Figure 1:** TGF-β facilitates EMT process and ECM deposition and downregulates miR-223-3p in EECs. (a) Wound healing assay for examining the migration of TGF-β-stimulated EECs. (b) Transwell assay for assessing the migratory and invasive abilities of TGF-β-stimulated cells. (c) Western blotting of EMT protein and ECM protein levels. (d) RT-qPCR analysis of miR-223-3p level in EECs treated with TGF-β. (e) RT-qPCR analysis of miR-223-3p level in IUA and normal tissues (*N* = 20 pairs). All experiments were performed in triplicate and data are presented as the mean value ± SD. Student’s *t*-tests were performed for statistical analysis. ***p < 0.001, TGF-β vs control group or IUA vs normal group.

### 3.2 miR-223-3p attenuates EMT process and ECM deposition

Subsequently, the impact of miR-223-3p in EECs was detected. Obviously, miR-223-3p level was raised after transfection of miR-223-3p mimics (Figure 2a). Next we applied TGF-β-stimulated EECs for the following assays. As shown by wound healing assay, cell migration was restrained by miR-223-3p mimics (Figure 2b). Likewise, Transwell assay revealed that miR-223-3p mimics suppressed cell migratory and invasive capabilities (Figure 2c). As displayed by western blotting, E-cadherin level was enhanced, while N-cadherin, Vimentin, α-SMA and collagen I levels were decreased in mimic-miR-223-3p group (Figure 2d). These revealed that miR-223-3p has a suppressive impact on EMT process and ECM deposition in EECs.

RETRACTED

**Figure 2:** MiR-223-3p alleviates EMT process and ECM deposition. TGF-β-treated EECs were used for the following assays. (a) RT-qPCR for detection of the transfection efficiency of miR-223-3p mimics. (b) Wound healing assay for detecting cell migration after overexpressing miR-223-3p. (c) Transwell assay for evaluating cell migration and invasiveness after transfection of miR-223-3p mimics. (d) Western blotting of EMT protein and ECM protein levels in miR-223-3p mimic group and the control group. All experiments were performed in triplicate and data are presented as the mean value ± SD. Student’s *t*-tests were performed for statistical analysis. **p < 0.01, ***p < 0.001, miR-223-3p vs NC mimics group.

### 3.3 miR-223-3p targets SP3

To figure out how miR-223-3p works in IUA, the downstream targets of miR-223-3p were predicted by miRDB (http://mirdb.org/cgi-bin/search.cgi). Two potential mRNAs (FBXW7 and SP3) were singled out (Figure 3a). RT-qPCR and western blotting elucidated that SP3 expression at mRNA and protein levels were suppressed after overexpressing miR-223-3p in EECs, while FBXW7 expression was almost unchanged (Figure 2b and c). TargetScan confirmed the existence of the complementary site of miR-223-3p on SP3 (Figure 3d). Furthermore, a luciferase reporter assay indicated that miR-223-3p mimics weakened the luciferase activity of SP3-Wt rather than SP3-Mut in EECs (Figure 3e). Collectively, SP3 is targeted by miR-223-3p. Furthermore, SP3 level in the endometrial tissues was detected. As shown by the results, SP3 was highly expressed in IUA in comparison to the control group (Figure 3f). Additionally, Pearson correlation analysis displayed that miR-223-3p and SP3 expression was negatively correlated in IUA tissues (*N* = 20) (Figure 3g).

**Figure 3:** MiR-223-3p targets SP3. (a) MiRDB was used for predicting downstream targets of miR-223-3p. (b) The mRNA levels of FBXW7 and SP3 in transfected-EECs analyzed by RT-qPCR. (c) Protein levels of FBXW7 and SP3 in EECs after overexpressing miR-223-3p detected by western blotting. (d) TargetScan was used for predicting the complementary site of miR-223-3p on SP3 3′UTR. (e) A luciferase reporter assay for detecting the association between SP3 3′UTR and miR-223-3p in EECs. (f) RT-qPCR analysis of SP3 level in IUA and normal tissues (*N* = 20 pairs). (g) Pearson analysis for analyzing the correlation between miR-223-3p and SP3 expression in IUA tissues (*N* = 20). All experiments were performed in triplicate and data are presented as the mean value ± SD. Student’s *t*-tests were performed for statistical analysis. ***p < 0.001, miR-223-3p vs NC mimics group or IUA vs normal group.

RETRACTED

### 3.4 SP3 upregulation rescues the suppressive impact of miR-223-3p mimics on the malignant phenotypes of EECs

Rescue assays were implemented to further identify the relationship between SP3 and miR-223-3p in IUA. We first tested the transfection efficiency of pcDNA3.1/SP3 by western blotting (Figure 4a). Moreover, wound healing assay displayed that the number of migratory cells reduced by miR-223-3p mimics were then increased by overexpressing SP3 (Figure 4b). In parallel, the suppressive impact of miR-223-3p on cell migration and invasiveness was offset by SP3 upregulation (Figure 4c). The miR-223-3p mimics-induced enhancement in E-cadherin level as well as reduction in N-cadherin, Vimentin, α-SMA and collagen I levels were reversed by pcDNA3.1/SP3, as revealed by western blotting (Figure 4d). In summary, SP3 can counteract the influence of miR-223-3p in IUA.

**Figure 4:** SP3 counteracts the influence of miR-223-3p. (a) Western blotting for analyzing pcDNA3.1/SP3 transfection efficiency. (b) Wound healing assay for evaluating cell migration after transfection of miR-223-3p mimics, miR-223-3p mimics + pcDNA3.1/SP3 or NC mimics. (c) Transwell assay for assessing the migration and invasion of EECs with above transfection. (d) Protein levels of EMT and ECM markers by western blotting in cells with above transfection. All experiments were performed in triplicate and data are presented as the mean value ± SD. Student’s *t*-tests were performed for panel (a), while ANOVA followed by Tukey’s *post hoc* analysis was performed for panels (b–d). *p < 0.05, **p < 0.01, miR-223-3p + SP3 vs miR-223-3p group; ***p < 0.001, SP3 vs vector group or miR-223-3p vs NC mimics group.

## 4 Discussion

A great number of studies have verified that miRNAs are abnormally expressed to regulate the cellular process in many diseases [28,29]. Recently, miR-223-3p has gained much attention and has been reported to implicate in inhibiting or promoting the fibrosis in some diseases. For example, miR-223-3p is sponged by circ_0070963 and targets LEMD3 to inhibit liver fibrosis [30]. miR-223-3p alleviates the progression of fibrosis and chronic inflammation in nonalcoholic steatohepatitis [31]. Furthermore, a previous study has confirmed that TGF-β stimulation enhances the expression of miR-223-3p in benign prostatic hyperplasia epithelial cells [23]. In our study, we investigated the impact of TGF-β in EECs. As revealed by the results, TGF-β acted as a motivator in cell migration and invasion. Similarly, TGF-β induced EMT process and ECM deposition in EECs. Contrary to the previous study [23], TGF-β stimulation was found to inhibit miR-223-3p expression. It was found that miR-223-3p was downregulated in IUA tissues compared to that in the normal samples. Additionally, miR-223-3p showed a suppressive impact on cell migration, invasion, EMT process and ECM deposition, suggesting an opposite effect of TGF-β. It has been clarified that EMT process and ECM deposition are positively related to endometrial fibrosis, the most important pathological feature of IUA [15,32,33]. Thus, based on these results, it can be summarized that TGF-β induces EMT process and ECM deposition, leading to endometrial fibrosis and subsequently the formation of IUA, and miR-223-3p can alleviate this impact.

RETRACTED

Subsequently, we analyzed how miR-223-3p exerts its effect on IUA. Numerous studies have demonstrated that miRNAs regulate gene expression by inhibiting transcription or driving degradation of downstream targeted mRNAs [34,35]. Based on bioinformatics analysis and the assays, we finally confirmed SP3 to be targeted by miR-223-3p. Results showed that SP3 was highly expressed in IUA tissues, and its expression was inversely correlated with miR-223-3p expression in the endometrial tissue samples. SP3 has been reported to interact with certain miRNAs to influence the development of human diseases. For example, miR-223 indirectly facilitates ATP-binding cassette transporter A1 expression by SP3 to regulate cholesterol homeostasis [36]. However, the interaction between miR-223-3p and SP3 in IUA has not been illustrated. In the present study, SP3 was found to reverse the influence of miR-223-3p. The rescue experiments suggested that SP3 attenuated the suppressive impact on the migration, invasion, EMT process as well as ECM deposition of EECs caused by miR-223-3p upregulation. The results suggested that miR-223-3p exerts its regulatory function in IUA by interacting with SP3.

In conclusion, we investigated the function and mechanism of miR-223-3p in IUA and discovered that miR-223-3p alleviated TGF-β-induced cell migration, invasion, EMT process and ECM deposition in IUA. Furthermore, miR-223-3p exerted above effect on EECs by targeting SP3. These findings might help to develop a novel therapeutic target for preventing IUA formation.
